The article "Correlation Analysis of Computed Tomography Features and Pathological Types of Multifocal Ground-Glass Nodular Lung Adenocarcinoma" was published in 2022. Journal: Comput Math Methods Med.

# Correlation Analysis of Computed Tomography Features and Pathological Types of Multifocal Ground-Glass Nodular Lung Adenocarcinoma

**DOI:** 10.1155/2022/7267036

**Published:** 2022-07-26

**Authors:** Jieli Kou, Xiaofei Gu, Liqing Kang

**Affiliations:** ^1^Graduate School, Tianjin Medical University, Tianjin 300070, China; ^2^Medical Imaging Center, Cangzhou People's Hospital, Cangzhou 061000, China; ^3^Department of Magnetic Resonance Imaging, Cangzhou Central Hospital, Cangzhou 061014, China

## Abstract

To investigate the correlation between computed tomography (CT) image characteristics of multiple lung ground-glass nodules (GGNs) and pathological classification, the CT image data of multiple lung GGN patients confirmed by pathology (*n* = 132) in our hospital were collected. The imaging features of GGNs were analyzed by qualified physicians, including lesion size (diameter, volume, and mass), location, CT values (mean and relative CT values), lesion morphology (round and irregular), marginal structure (pagination and burr), internal structure (bronchial inflation sign), and adjacent structure (pleural depression). CT imaging analysis was performed for the subtype of infiltrating adenocarcinoma (IAC). In CT findings, GGNs were greatly different from adenomatous hyperplasia (AAH), pure GGN adenocarcinoma in situ (AIS), and microinvasive adenocarcinoma (MIA) in terms of marginal structure, lesion morphology, internal structure, adjacent structure, and size (*P* < 0.05). The mean and relative CT values of mural adenocarcinoma, acinar adenocarcinoma, and papillary adenocarcinoma of IAC subtypes were greatly different from those of AAH/AIS/MIA (*P* < 0.05). In summary, the CT images of GGNs can be used as the basis for the differentiation of AAH, AIS, and MIA early noninvasive types and IAC invasive types, and the CT value of the IAC subtype can be used as the basis for the classification and differentiation of IAC pathological subtypes.

## 1. Introduction

Lung cancer is a relatively common malignant tumor with the highest morbidity and mortality throughout the year [1]. Although smoking is the main risk factor accounting for 80% to 90% of all lung cancer diagnoses [2], in recent years, the incidence among young and nonsmoking people has also shown an increasing trend, posing a serious threat to the health of Chinese people [3]. Lung cancer can be mainly classified into non-small-cell lung cancer (NSCLC) and small-cell lung cancer (SCLC). Among all lung cancers, NSCLC accounts for approximately 85-88%, and SCLC accounts for approximately 12-15% [4]. NSCLC is classified into three types according to its characteristics and treatment measures, namely, adenocarcinoma (55%), squamous cell carcinoma (35%), and large cell carcinoma (10%) [5]. The probability of malignancy varies with the density of pulmonary nodules. Pulmonary nodules are classified into three types according to density, namely, ground-glass nodules (GGNs), solid nodules (SNs), and partial solid nodules (PSNs) [6]. The malignant probability from high to low is partially solid nodules, GGNs, and solid nodules [7].

The article "Correlation Analysis of Computed Tomography Features and Pathological Types of Multifocal Ground-Glass Nodular Lung Adenocarcinoma" was published in 2022. Journal: Comput Math Methods Med.

GGN refers to the fuzzy nodules in the lung. The density of nodules is slightly higher than that of the surrounding lung parenchyma, but the outline of blood vessels and bronchus within the nodules can be seen [8]. Causes of GGN include inflammation, pulmonary fibrosis, and the most common early lung adenocarcinoma [9]. The study found that simple GGNs gradually evolved into lung adenocarcinoma (LA) during long-term follow-up, and lung adenocarcinoma was classified into atypical adenomatous hyperplasia (AAH), adenocarcinoma in situ (AIS), minimally invasive adenocarcinoma (MIA), and invasive adenocarcinoma (IAC) [10]. Lung adenocarcinoma is more likely to metastasize earlier than lung squamous cell carcinoma, so lung adenocarcinoma has a poor prognosis and needs early diagnosis and treatment [11]. The pathological degree of early GGN was sorted according to the degree of malignancy, degree of invasion, and prognosis. AAH had the smallest volume, the lowest surgical trauma, and the lowest degree of malignancy, and the prognosis was the best without considering complications. Sometimes, after long-term observation, it is found that AAH does not change much and does not require treatment [12]. AIS has basically no difference in size compared with AAH, and the degree of malignancy is poor. Some lesions are slightly infiltrated, so they are difficult to identify, and the prognosis is better than that of MIA [13]. MIA is mainly mural growth, and the pathological differentiation between MIA and IAC mainly includes invasion of blood vessels and lymphatics, invasion of the pleura and airway, tumor necrosis, and airway transmission [14]. IAC is the final stage in the transformation of lung cancer, and there are five subtypes, namely, apical, acinar, papillary, solid, and micropapillary. The adherent type corresponds to high differentiation, acinar and papillary types correspond to medium differentiation, and solid and micropapillary types correspond to low differentiation. The higher the degree of differentiation, the better the prognosis, and the higher the proportion of the micropapillary type and solid type, the worse the prognosis.

After the widespread use of low-dose computed tomography (CT) in lung cancer examination, the number of GGNs detected has increased. Preoperative detection and positioning of GGNs by CT to identify the subtypes of early lung adenocarcinoma is crucial for accurate preoperative pathological diagnosis of patients by clinical staff [15]. However, how to distinguish infiltrating lesions from non- or microinfiltrating lesions according to CT images and enable patients to receive surgical treatment as soon as possible is the research focus of radiologists. The CT features of GGNs are related to the pathology of lung adenocarcinoma GGNs. With the development and popularization of high-resolution computed tomography (HRCT), the positional relationship between GGNs and surrounding capillaries and bronchi can be clearly displayed [16]. HRCT has obvious application value in the identification of GGNs and makes it possible to determine the pathological subtypes of lung adenocarcinoma with the CT features of GGNs. Clinicopathological diagnosis is the gold standard for differentiating cancer, and no CT, MRI, or other examination can ultimately determine the nature and type of lesions. Therefore, the study of the relationship between CT examination and pathological diagnosis is helpful to continuously improve the diagnostic accuracy of clinicians [17]. At present, there is no unified diagnostic standard for CT diagnosis of GGNs in clinical practice. In this study, the CT image features of GGNs were analyzed to distinguish different pathological subtypes of IAC and to study the relationship between the CT features of GGNs and pathological types of lung adenocarcinoma.

The article "Correlation Analysis of Computed Tomography Features and Pathological Types of Multifocal Ground-Glass Nodular Lung Adenocarcinoma" was published in 2022. Journal: Comput Math Methods Med.

## 2. Materials and Methods

### 2.1. General Information

In this study, 132 patients with chest CT examination and pathologically confirmed GGNs in hospital from May 2020 to May 2021 were enrolled. Inclusion criteria are as follows: complete and clear preoperative CT images of patients can be harvested through picture archiving and communication system (PACS); there were at least two GGNS with maximum diameters of no less than 25 mm in both lungs; postoperative pathology required thoracoscopic or thoracoscopic resection and staining, which was reviewed by at least one senior pathologist with 10 years of experience in diagnosis of tumor pathology, and pathological subtypes were classified according to the new classification in 2015. Exclusion criteria are as follows: patients unable to undergo surgical treatment and patients with incomplete imaging data. At the beginning of this study, patients or their families signed informed consent. This study was approved by the ethics committee of the hospital.

### 2.2. Examination Methods

64-slice spiral CT machine was employed. Breath-holding training was performed before scanning, and the breath-holding state under breathing was calm during scanning. The supine position was the dominant position, and some patients were in the prone position. First, the whole lung was scanned with a thickness of 5-10 mm, including the axilla and chest wall on both sides. After GGN was found, a CT scan was performed again. The layer thickness was 1.25 mm target scan, and the standard algorithm and bone algorithm were reconstructed. The target scanning parameters were as follows. The collimator was 1.25 mm, the pitch was 1.375, the tube voltage was 120 kV, the tube current was 250-350 mAs, the field of vision was 16-24 cm, and the matrix was 512 × 512. MPR was performed on all patient raw data at a 1.25 mm layer thickness on an ADW 4.5 or 4.7 workstation. The accompanying signs of GGN were displayed, with emphasis on the walking, morphology, and lumen of the relevant bronchi, and the relationship between them and lesions was recorded.

The article "Correlation Analysis of Computed Tomography Features and Pathological Types of Multifocal Ground-Glass Nodular Lung Adenocarcinoma" was published in 2022. Journal: Comput Math Methods Med.

### 2.3. CT Scanning and Image Processing

The images were analyzed separately by two highly qualified physicians in the Department of Radiology, and the results were statistically analyzed. If there was any deviation in the analysis, the consensus of the two physicians was taken as the result.

### 2.4. Evaluation Content

The evaluation included location (right upper lobe, right middle lobe, right lower lobe, left upper lobe, and left lower lobe), lesion morphology (round and irregular), marginal lobulation and burr, internal structure (air bronchial sign), bronchial truncation, adjacent structure (pleural depression), lesion size (diameter and volume and mass), mean CT value, and relative CT value. Diameter was the average diameter of GGN, that is, the average of long diameter + short diameter on the largest layer of GGN in CT images. The maximum layer length *L*, short diameter *W*, and thickness *T* (number of nodular layers × layer thickness) of GGNs were calculated, and the volume was calculated according to Equation (1). The mass was calculated according to Equation (2) [18].

(1) $$\begin{array}{c} V=\frac{1}{6}\pi \times L\times W\times T, \end{array}$$

(2) $$\begin{array}{c} g=\frac{V\times \left(1000+\text{CT value}\right)}{10^{6}}. \end{array}$$

The average CT value was measured at the corresponding GGN position three times and averaged. The relative CT value was the ratio of the average CT value of the largest layer of GGNs in the CT lung window to the average CT value of normal lung tissue in the same plane. When the GGN looks like a wave or shell edge, it is called a leaf-splitting sign. The burr mark is a nodular shadow with tubercle margins not reaching the pleura. Vacuolar sign refers to small round vacuoles appearing in nodules, while bronchial aeration sign refers to GGN signs containing gas in bronchioles that cross nodules. Therefore, it is difficult to distinguish between the two images, so the experiment was combined with statistics.

The article "Correlation Analysis of Computed Tomography Features and Pathological Types of Multifocal Ground-Glass Nodular Lung Adenocarcinoma" was published in 2022. Journal: Comput Math Methods Med.

### 2.5. Postoperative Pathological Analysis

After surgical resection, the lesions were fixed with paraformaldehyde and embedded in paraffin. Hematoxylin-eosin staining and immunohistochemical staining were performed after sectionalization. Classification and classification statistics were carried out according to the pathological classification method of lung adenocarcinoma subtype published by the World Health Organization (WHO) in 2015 [19].

### 2.6. Statistical Methods

SPSS 22.0 was used for data processing. ANOVA was used for measurement data. The Kruskal–Wallis *H* test was used when the samples did not conform to a normal distribution. The *χ*^2^ test was used for technical data. *P* < 0.05 indicated that the difference was statistically significant.

## 3. Results

### 3.1. Statistical Results of Clinical Data

The patients were divided into two groups according to the degree of invasion. Sixty-seven patients had preinvasive lesions of lung adenocarcinoma (AAH/AIS/MIA group). There were 65 patients with infiltrating adenocarcinoma (IAC group). In the IAC group, there were three subtypes, including 38 cases of adherent growth type IAC, 18 cases of acinar IAC, and 9 cases of papillary IAC. The clinical data of all GGN cases are shown in Table 1. The age of patients with IAC was higher than that of AAH, AIS, and MIA, and the difference was statistically significant (*P* < 0.05). The data of various pathological subtypes of IAC are shown in Table 2, and there was no significant difference between the data of various pathological subtypes of IAC (*P* > 0.05).

### 3.2. GGN Site Statistics Result

In Figure 1, there was no significant difference in GGN location between the AAH/AIS/MIA group and the IAC group (*P* > 0.05). There was no significant difference in the location of each pathological subtype of IAC (*P* > 0.05).

### 3.3. GGN Margin and Lesion Morphology

In Figure 2, the comparison of noninvasive and invasive GGN margins found that the number of GGNS with pagination and burrs in IAC margins was much higher than that in AAH/AIS/MIA (*P* < 0.05), and there was no significant difference among IAC subgroups. Comparison of noninvasive and invasive GGN lesions showed no significant difference between IAC and AAH/AIS/MIA or between IAC subgroups.

### 3.4. GGN Internal Structure and Adjacent Structure

Since the bronchial inflation sign and air bubble sign are not easy to judge, both were counted as bronchial inflation signs in this experiment. In Figure 3, the number of bronchial inflation signs and pleural depression signs in IAC was much higher than that in AAH/AIS/MIA, and the difference was statistically significant (*P* < 0.05). There were no significant differences among the IAC subgroups.

The article "Correlation Analysis of Computed Tomography Features and Pathological Types of Multifocal Ground-Glass Nodular Lung Adenocarcinoma" was published in 2022. Journal: Comput Math Methods Med.

### 3.5. Diameter, Volume, and Mass of GGNs

In Figure 4, the diameter, volume, and mass of infiltrating GGNs were much higher than those of noninfiltrating GGNs, and the difference was statistically significant (all *P* < 0.05). There was no significant difference between IAC subtypes (all *P* > 0.05).

### 3.6. Mean and Relative CT Values

In Table 3, both CT values and relative CT values of pathological subtypes in the IAC group were significantly different from those in the noninvasive AAH/AIS/MIA group (*P* < 0.05).

### 3.7. CT Features and HE Staining Analysis of GGNs

Atypical adenoma hyperplasia (Figure 5(a)) is a benign hyperplastic disease that is also considered a precancerous lesion and may become cancerous if left untreated. Atypical adenomatous hyperplasia is a millimeter micronodular lesion that is indistinguishable from normal lung tissue in color and texture. It occurred in the central area of the acinar near the respiratory bronchioles and consisted of mild-to-moderate atypia of type II alveolar cells or Clara cells growing along the alveolar wall (Figure 5(i)), which can form inconspicuous pseudopapillae. Nonmyxoid AIS showed nonsolid ground glass shadows (Figure 5(b)), which was histologically similar to atypical adenomatous hyperplasia. The tumor cells in situ were denser, crowded, and lacked intercellular spaces (Figure 5(j)). Mucinous in situ adenocarcinoma often presents as solid nodules. Tall columnar tumor cells grow adherents with nuclei in the basement and a large amount of mucus in the cytoplasm (Figure 5(k)), similar to goblet cells, and the nuclei may be completely free of atypia. Chest CT of an MIA showed a small and impure GGN (Figure 5(c)) with a growth pattern other than adherence infiltrating into the stroma containing myofibroblasts (Figure 5(l)). Infiltrating adenocarcinoma presented irregular nodular shadows accompanied by vascular cluster signs and pleural depression signs (Figure 5(d)). Generally, HE staining (Figure 5(e)) showed three different subtypes, namely, the papillary type (Figure 5(f)), acinar type (Figure 5(g)), and mural type (Figure 5(h)).

## 4. Discussion

Lung cancer is more insidious than other cancers, and once symptoms appear, it is basically at an advanced stage, so physical examination is an effective means to find early lung cancer. CT is the most commonly used method for the diagnosis of lung cancer at present, which also leads to the delayed early diagnosis of lung cancer, so early CT detection is crucial [20]. GGN, as a CT imaging manifestation of early lung cancer, has received increasing attention. However, low-dose CT also detected massive GGNs. Classification of GGNs and subtypes of lung adenocarcinoma cases by CT can help improve the accuracy of clinical staff's preoperative diagnosis of patients and select more accurate treatment methods for lesions [21]. The histological growth pattern and biological function of lung adenocarcinoma determine the gradual increase in density and change in morphology in the development process, so the manifestation on CT shows that GGN develops into PSN and SN.

The article "Correlation Analysis of Computed Tomography Features and Pathological Types of Multifocal Ground-Glass Nodular Lung Adenocarcinoma" was published in 2022. Journal: Comput Math Methods Med.

Pathological studies of lung cancer have found that the increase in density and size of lesions is often a symbol of malignant lesions, so the size, volume, and mass of lesions are correlated with the degree of malignancy of lesions [22]. Three-dimensional GGN statistics have good repeatability and are most sensitive to changes in GGN volume with high specificity. Therefore, the GGN quality calculated by the volume of GGN can also well reflect the volume and density changes of GGN, with stronger accuracy and objectivity, which is of great significance to evaluate the pathology of GGN [23]. Some studies have found that the higher the diameter and execution composition of GGNs are, the higher the degree of malignancy of the tumor [24]. This study also found that the diameter, volume, and mass of IAC infiltrating lesions were much higher than those of noninfiltrating lesions, and the differences were statistically significant. The morphology of GGNs showed that the pagination morphology of IAC lesions was higher than that of noninvasive lesions, and the difference was statistically significant. The main reason for this phenomenon is the diversity of cell growth in GGNs with different growth rates. Some cells with faster growth rates are blocked by adjacent lung tissues or interstitium, resulting in growth restriction and lobular signs [25]. Vacuolar or bronchoinflated signs appear histologically because tumor cells spread along the lung interstitium and the bronchial wall, mainly in the form of mural growth. This growth mode is more likely to invade the alveolar structure and fuse with the alveolar or bronchial wall to form an air cavity [26]. The number of cases with vacuolar or bronchoinflated signs of IAC was greater than that of non-IAC, and the difference was statistically significant. The pleural depression sign lesion was close to the pleura, and there was a contractile force, resulting in the adjacent pleura being pulled so that it was pulled to the side of the lesion. The occurrence of pleural depression indicates that the degree of malignancy of tumors is generally high. In this study, it was also found that the incidence of pleural depression in IAC infiltrating lesions was significantly higher than that in noninfiltrating lesions. In addition, the age of patients with AAH/AIS/MIA noninvasive surgery was lower than that of patients in the IAC group. This may be related to the pathological development of GGNs. The younger the patients are, the more benign the pathological type of GGN, while the older the patients are, the more likely the GGN pathology is malignant [27]. The progression of CT imaging manifestations of GGNs from AAH to IAC also means an increase in the execution components, density, and CT value, which also suggests the progression trend of pathological types of the lesions. This in turn explains why the age of onset in the IAC group was older than that in the preinvasive or MIA group. In general, the more real components of the GGN, the higher the CT value. This study found that the average CT value of each subgroup with IAC infiltration was higher than that of AAH/AIS/MIA, and the difference was statistically significant. This is related to the higher proportion of GGN solid components in each pathological subtype. The subtypes of IAC, if ordered by mean CT value, were found to have the lowest mean CT value in the mural growth type and vascular or lymphatic invasion. There was less pleural invasion or cellular airway spread or necrosis, and the average CT value of acinar type IAC was lower than that of papillary type. In addition, papillary IAC is more prone to vascular invasion or lymphatic invasion, pleural invasion, or cellular airway spread or necrosis, especially the airway spread of tumor cells, due to its histological morphology [28, 29].

The article "Correlation Analysis of Computed Tomography Features and Pathological Types of Multifocal Ground-Glass Nodular Lung Adenocarcinoma" was published in 2022. Journal: Comput Math Methods Med.

## 5. Conclusion

In this study, CT features and pathological features of multiple GGN were used to explore the correlation between the two. It was found that the imaging features of GGN could be used as a reliable basis for the identification of AAH, AIS, MIA, and IAC, which were especially effective in the features of GGN's edge structure, lesion morphology, internal structure, adjacent structure, and size. The pathological subtypes of IAC can be distinguished by the mean CT value and relative CT value in early noninvasive lung adenocarcinoma of AAH, AIS, and NIA. However, the deficiency of this study is that the number of patient samples is small, which cannot reflect the actual situation more objectively. More experimental cases should be included in subsequent studies. In addition, follow-up was not considered in this retrospective study, and multiple GGNS proved to be atypical adenomatous hyperplasia, AIS, microinvasive adenocarcinoma, and invasive adenocarcinoma after thoracoscopic or thoracotomy resection was included. The included samples were somewhat deviated, and isolated GGNS were not considered. In conclusion, this study is helpful for surgeons and radiologists to distinguish between patients with invasive and noninvasive lesions before surgery and to adopt different treatment regimens to improve patient outcomes.

## Figures and Tables

**Figure 1:** GGN location statistics. a–f showed the GGN location statistics of the upper lobe of the right lung, middle lobe of the right lung, lower lobe of the right lung, upper lobe of the left lung, lower lobe of the left lung, and various pathological subtypes of IAC, respectively.

**Figure 2:** The marginal condition and lesion morphology of GGNs. (a–d) The pagination and burr at the edges of noninvasive GGNs and invasive GGNs, edge morphology of each pathological subtype of IAC, round and irregular lesion morphology of noninvasive GGNs and invasive GGNs, and lesion morphology of each pathological subtype of IAC, respectively. ^∗^Compared with the noninfiltrating AAH/AIS/MIA group, *P* < 0.05.

**Figure 3:** GGN internal structure and adjacent structure statistics. (a–d) The number of bronchial inflation signs in noninvasive GGNs and invasive GGNs, the internal structure of each pathological subtype of IAC, the number of noninvasive and invasive GGNs whose adjacent structures were pleural depressions, and the statistical analysis of adjacent structures of various pathological subtypes in IAC, respectively. ^∗^Compared with the noninfiltrating AAH/AIS/MIA group, *P* < 0.05.

**Figure 4:** Diameter, volume, and mass statistics of GGNs. (a–f) The diameter of the noninfiltrating type and infiltrating type GGN, diameter of each pathological subtype of IAC, volume of the noninfiltrating type and infiltrating type GGN, volume of each pathological subtype of IAC, mass of the noninfiltrating type and infiltrating type GGN, and mass of each pathological subtype of IAC, respectively. ^∗^Compared with the noninfiltrating AAH/AIS/MIA group, *P* < 0.05.

**Figure 5:** CT features of different GGNS and HE staining of infiltrating lung adenocarcinoma. (a) A CT scan of atypical adenomatous hyperplasia in the lower lobe of the patient's left lung; (b) a CT scan of a pure GGN in situ adenocarcinoma in the upper lobe of the patient's right lung; (c) an MIA in the middle lobe of the patient's right lung; (d) an invasive adenocarcinoma in the lower lobe of the patient's right lung; (e) the HE ×200 staining diagram of invasive lung adenocarcinoma; (f) the HE ×200 staining diagram of papillary lung adenocarcinoma; (g) the HE ×100 staining diagram of acinar lung adenocarcinoma; (h) the HE ×100 staining diagram of mural lung adenocarcinoma; (i) the HE ×200 staining of atypical cell lung cancer; (j) the HE ×100 staining of nonmucinous in situ lung adenocarcinoma; (k) the HE ×200 staining of mucinous in situ lung adenocarcinoma; (l) the HE ×100 staining of MIA.

The article "Correlation Analysis of Computed Tomography Features and Pathological Types of Multifocal Ground-Glass Nodular Lung Adenocarcinoma" was published in 2022. Journal: Comput Math Methods Med.

**Table 1:** Clinical data information of patients.

GGN type	Cases	Age	Sex	
			Male	Female
AAH	19	46.14 ± 5.78	10	9
AIS	23	46.01 ± 6.02	13	10
MIA	25	45.34 ± 5.14	12	13
IAC	65	51.76 ± 4.99^∗^	29	36

^∗^Compared with the noninfiltrating AAH/AIS/MIA group, *P* < 0.05.

**Table 2:** Clinical data of IAC subtype.

IAC subtype classification	Cases	Age	Sex	
			Male	Female
Adherent growth IAC	38	51.72 ± 4.99	18	20
Acinar IAC	18	50.01 ± 5.06	8	10
Papillary IAC	9	51.66 ± 5.18	3	6

**Table 3:** Comparison of mean and relative CT values between the infiltrating IAC group and the noninfiltrating AAH/AIS/MIA group.

Type	AAH/AIS/MIA	Pathological subtypes of IAC		
		Adherent growth IAC	Acinar IAC	Papillary IAC
CT value (HU)	−651 ± 103	−603 ± 76^∗^	−589 ± 89^∗^	−565 ± 73^∗^
Relative CT value (HU)	0.77 ± 0.05	0.63 ± 0.12^∗^	0.65 ± 0.11^∗^	0.53 ± 0.14^∗^

^∗^Compared with the AAH/AIS/MIA group, *P* < 0.05.

## Data Availability

The data used to support the findings of this study are available from the corresponding author upon request.
